The article "Postoperative Effects of Dexmedetomidine on Serum Inflammatory Factors and Cognitive Malfunctioning in Patients with General Anesthesia" was published in 2021. Journal: J Healthc Eng.

# Postoperative Effects of Dexmedetomidine on Serum Inflammatory Factors and Cognitive Malfunctioning in Patients with General Anesthesia

**DOI:** 10.1155/2021/7161901

**Published:** 2021-09-07

**Authors:** Zitan Zhang, Wei Li, Huiqun Jia

**Affiliations:** ^1^Department of Anesthesiology, The Fourth Hospital of Hebei Medical University, 12 Jiankang Road Shijiazhuang, Hebei 050011, China; ^2^Department of Anesthesiology, The Second Hospital of Hebei Medical University, 215 Heping West Road Shijiazhuang, Hebei 050000, China

## Abstract

**Objective:**

To investigate the effects of dexmedetomidine intervention on serum inflammatory factor concentration and postoperative cognitive malfunction in elderly patients with general anesthesia. *Methodology*. 174 patients with general anesthesia were selected, who were categorized into a control group (HC) and a dexmedetomidine group (HS) using the random number table method, with 87 patients in individual groups. The dexmedetomidine group was pumped intravenously with dexmedetomidine at a loading dose of 1 *μ*g/kg before induction of anesthesia for 15 min, followed by continuous intravenous pumping at a rate of 0.4 *μ*g/kg/h, and the dosing was stopped at 30 min before concluding the surgery. The control group was administered the identical dose of saline in the same manner. Interleukin 6 (IL-6) and tumor necrosis factor *α* (TNF-*α*) levels and MMES scores were tested at 1 h before and 24 h after anesthesia.

**Results:**

Comparing to HC group, patients in the HS group had lower TNF-*α* and IL-6 levels at both scheduled points (*P* < 0.05).

**Conclusion:**

Dexmedetomidine reduced the expression of inflammatory factors in elderly patients with general anesthesia and effectively reduced the incidence of postoperative cognitive dysfunction after general anesthesia surgery.

## 1. Introduction

Postoperative cognitive dysfunction (POCD) has a high incidence in elderly patients undergoing general anesthesia, and there is still no clear pathogenesis. It is generally believed that POCD refers to a group of complications of the patient's central nervous system (CNS) after anesthesia surgery. Its formation mechanism is complex, which may be related to age, surgery type, and anesthetic type [1]. It is more common in elderly patients, manifesting as impairment in patients' memory, attention, learning ability, abstract thinking, and orientation. Most are accompanied by a decrease in the ability to adapt to society, to interact with others, and to perform daily activities. It often lasts for several days, with a few lasting for several weeks. POCD has become a common and frequent disease in the elderly after surgery. With the development of economy and society, Chinese society is rapidly entering the aging society. Therefore, strengthening the research on POCD is in line with the trend of social development and has significant socioeconomic significance.

The neuroinflammatory mechanism is one of the most important theories in the current mechanistic studies. Neuroinflammation is mostly caused by systemic inflammation, and the body causes central nervous system inflammation through different pathways and mechanisms, leading to constructional and functional alterations in the central nerve cells, resulting in POCD. The main view is that POCD is a neurological disorder induced by surgical and anesthesia-induced changes in the structure of central nerve cells in elderly patients based on degenerative changes in the brain and preexisting diseases in other organs and systems of the body. Since POCD is a kind of central nerve injury, clinical anesthesia needs to find a drug that can protect the central nerve and suppress the inflammatory response. Dexmedetomidine (DEX) is one of the most recently studied anesthetic adjuncts that can protect organ function by decreasing the release of sympathetic ganglion fiber neurotransmitters, thereby reducing the production of related inflammatory factors, and by inhibiting oxidative stress and reducing reperfusion injury. This study was conducted to try to understand the relationship between inflammatory factors, dexmedetomidine, and postoperative cognitive dysfunction by preoperative- and postoperative-related inflammatory factors in patients undergoing general anesthesia.

## 2. Materials and Methods

A total of 174 elderly patients scheduled for surgery with ASA grade I–III from January 2018 to June 2019 were selected. Among them, there were 75 patients with lumbar disc herniation, 36 prostatectomy patients, 31 cholecystectomy patients, and 6 patients with radical rectal cancer. These patients were randomized into two categories: the “dexmedetomidine group” and the “saline control group.” Eighty-seven patients were included in the dexmedetomidine group, 56/32 males/females of 61–89 years of age with mean age of 70.6 ± 4.2 years; body weight was 45–95 Kg with mean weight of 65.8 ± 5.8 kg. Education outlined was illiterate 11, primary 21, secondary 35, and above secondary 20, respectively. A total of 31 cases were classified as ASA grade I, 47 cases as ASA grade II, and 9 cases as ASA grade III. The control group included 87 patients, 58 males and 19 females from 61 to 92 years of age with 71.4 ± 4.9 mean age and body weight 47–94 kilograms with 66.2 ± 5.5 mean weight. Education outlined was illiterate 8, primary 16, secondary 23, and above secondary 14, respectively. A total of 22 cases were classified as ASA grade I, ASA grade II had 32 cases, and ASA grade III had 7 cases. Reportedly, the two groups had no statistically significant difference in general information such as age and gender (*P* > 0.05), and they were comparable (Table 1).

### 2.1. Inclusion and Exclusion Criteria

Inclusion criteria: patients with 18–79 years of age; ASA grade I–III; operation time within 24 hours; preoperative approval by the ethical board committee and voluntary signing of the study consent form. Exclusion criteria: those with a history of dementia and psychosis; those with severe cerebrovascular disease; those with a history of multiple surgeries; those with a history of severe perioperative infections in various systems; those with perioperative massive hemorrhage and severe acid-base imbalance and electrolyte imbalance; those with diabetes mellitus; and those with perioperative hormone.

### 2.2. Experimental Protocol

All patients were fasted for 8 h and dehydrated for 2 h before surgery, and no drugs were administered before surgery. After entering the operating room, peripheral veins were routinely opened and patients' heart rate, blood pressure, oxygen saturation, and EEG dual-frequency index were monitored, and internal jugular venipuncture and radial artery puncture were conducted after anesthesia induction to monitor patients' central venous pressure and invasive arterial pressure. Anesthesia method: sufentanil 0.4 *μ*g/kg, propofol 1 mg/kg, midazolam 0.05 mg/kg, and cis-atracurium 0.3 mg/kg were injected intravenously for anesthesia induction and wind pipe (tracheal tube) was inserted after 5 min. The anesthesia machine was connected for mechanical ventilation after determining the correct position of the tracheal tube, with VT 8–10 mL/kg, RR 12–16 times/min, and IE 1 : 2. PETCO_2_ was maintained at 35–40 mmHg and FiO_2_ at 60%. Anesthesia was maintained by inhalation of sevoflurane at concentrations of 1% to 2% and intravenous infusion of ∼6 mg/kg/h of propofol , 0.1∼0.5 *μ*g/kg/min remifentanil, and 0.1∼0.2 mg/kg/h cis-atracurium. The intraoperative inhaled concentration of sevoflurane was regulated according to the hemodynamic and BIS values, maintaining a BIS value of 40 to 60. Narcotic analgesics and vasoactive drugs were used so that the intraoperative BP and HR fluctuations did not exceed 20% of the basic value, and the mean value of arterial pressure must not be below 60 mmHg. If the fluctuation of BP and HR was greater than 20% of the preoperative base value, a comprehensive analysis and judgment would be made by using the depth of anesthesia monitor, and the specific intervention was to add 5 *μ*g of sufentanil and 0.3 mg of atropine or 2 *μ*g of norepinephrine each time and dexmedetomidine loading dose 1 *µ*g/kg was administered intravenously for 10 min, which were all monitored until medications took effect and vital signs returned to stability. When the adverse reaction of dextrometomidine happened, such as hypotension, hypertension, nausea, bradycardia, and dry mouth, the infusion was immediately discontinued. Over the next 24 hours, patients receiving the drug were closely monitored. After surgery and anesthesia, the patient was transferred to the postanesthesia recovery unit for resuscitation. All procedures were performed by the same group of physicians.

### 2.3. Examination Indicators and Methods

A total of 4 mL of elbow venous blood was collected before surgery (T1) and 24 h after surgery (T2), respectively, and centrifugation was performed to separate the serum. Enzyme-linked immunosorbent assay was used to detect the concentration of serum TNF-*α* and IL-6, in strict accordance with the instructions for use of the kit.

### 2.4. The POCD and Inflammatory Mediators Link Was Assessed by Quartiles

The values of TNF-*α* and IL-6 were arranged from smallest to largest and the three quartiles (Q1, Q2, and Q3) were Ql = (87 + 1)/4 = 22, Q2 = 2^*∗*^(87 + 1)/4 = 44, and Q3 = 3^*∗*^(87 + 1)/4 = 66. These four individuals divided 87 patients into four segments (q1, q2, q3, and q4). A comparison was performed with the POCD number within this quartet intersegments and then the correlation between POCD and these two inflammatory mediators was evaluated using Pearson's correlation analysis.

### 2.5. Statistical Analysis

The extracted data were statistically analyzed by using statistical software SPSS 17.0 (SPSS Inc., Chicago, II). For numerical variables, *t*-tests were performed both with paired and independent samples. If the data values conformed to normality and chi-squaredness, otherwise, signed rank sum test and Kruskal–Wallis test were used. The chi-square test was used for categorical variables. Correlation analysis was expressed as Pearson correlation coefficient. The test level was *P* = 0.05.

## 3. Results

The incidence of POCD was calculated in both experimental and control groups as 9.20% and 21.31%, respectively. There was a statistically significant difference between both experimental and control groups (*P* = 0.038). The levels of IL-6 and TNF-*α* in both groups were significantly higher than before surgery (Table 2). The increase was significantly suppressed in the dexmedetomidine group comparing to the control group (*P* < 0.05). POCD occurrence was also analyzed and statistically significant difference was also reported between the odds, when the levels of inflammatory mediators were different in the quartile grouping (*P* < 0.05). The relationship between two inflammatory mediators and POCD was calculated by Pearson's correlation analysis, and the correlation coefficients were *R* = 0.689 for IL-6 and *P* = 0.043 for POCD and *R* = 0.711 and *P* = 0.038 for TNF-*α* and POCD (Table 3).

Table 4 shows that with the increase of TNF-*α* values, the number of POCD also increases significantly (*P* < 0.05).

The data from Tables 4 and 5 were analyzed by Pearson's correlation analysis, which showed that the serum value of IL-6 concentration was significantly correlated with the number of POCD, i.e., *r* = 0.689 and *P* = 0.043. Likewise, serum concentration of TNF-*α* was also significantly and positively linked with POCD, i.e., *r* = 0.711 and *P* = 0.038. *P* < 0.05, suggesting that the elevated concentrations of proinflammatory factors were correlated with POCD (Tables 4 and 5).

## 4. Discussion

Studies have shown that the POCD incidence in elderly individuals encountering noncardiac surgical procedure is up to 25.8% and 9.9% at 1 week and 3 months postoperatively [2]. POCD is a degenerative change in neurological function induced or aggravated by a combination of surgical, anesthetic, and preexisting diseases based on the degeneration of the central nervous system. Monk and Price [3] have confirmed that the occurrence of POCD not only prolongs hospitalization time and increases patients' hospital costs but also leads to neurological impairment.

Numerous factors influence POCD in clinical practice, such as patient age, gender, education level, type of surgery, anesthesia method, and medications [4]. In this trial, a randomized approach was used in the design regarding the abovementioned factors, and there were no statistically significant differences in age, education level, duration of surgical anesthesia, and intraoperative medication between the two groups in this study. Besides, BIS was used to maintain the same depth of anesthesia during the operation, so as to ensure the homogeneity of the study population.

In the mechanisms of POCD, the theory of inflammatory response of central nervous system has gradually become a research hotspot, and validation plays an important role in this process [5], where tissue damage due to surgery can activate the peripheral intrinsic immune system and cause inflammatory cell infiltration, which in turn releases inflammatory mediators (TNF-*α*, IL-6, IL-1, etc.) [6]. Inflammatory reactions of the central nerve system can be caused by peripheral inflammatory factors entering the central nervous system. Peripheral inflammatory factors can enter the central nervous system through the blood-brain barrier or synthesize and release inflammatory factors by activating neuroendocrine cells in the blood-brain barrier, causing central inflammation. Inflammatory factors entering the CNS interfere with neuronal activity, thereby disrupting intersynaptic connections and signaling [7]. It has been shown that the degree of increased expression of proinflammatory factors and its presence in the central nervous system and body circulation of surgical patients may correlate with the degree of cognitive decline [8,9]. Interleukin 6 plays an important role in body's defense mechanism, immune system, and generating inflammatory responses in vivo. It also affects the growth and differentiation of central nerve cells in the CNS, which also influence cerebral functionality, specifically learning, investigation, and recollection of memory. IL-6 is secreted by intracranial microglia, neuronal cells, and astrocytes and has been implicated in brain injury. Normal concentrations of IL-6 levels are important for neuronal cell protection and repair; however, if the concentrations are too high, they instead exacerbate neuronal and microglial cell damage [10]. These processes may include synaptic plasticity or neuronal cell growth regulation [11].

TNF-*α* is secreted by macrophages and has a wide range of biological activities with extremely important roles in immune body regulation, regulation of inflammatory responses, neuroendocrine regulation, and other systems. TNF-*α* is involved in many aspects of daily activities of life such as sleeping, eating, bathing, and other autonomous processes. Recent studies have found that it is involved in the processes of learning and memory and plays a vital role in the pathology of POCD. The mechanism may be related to the processes that affect synaptic shaping and inhibit the growth and differentiation of nerve cells [12]. After surgery, TNF-*α* is the first cytokine to be released, and it is the initiating and amplifying factor of the inflammatory cascade response. Animal studies have shown that peripheral TNF-*α* can cause neuronal inflammation and lead to cognitive decline by inducing the release of IL-1 in the brain [13]. The hippocampus-dependent cognitive decline induced by chronic neuronal inflammation can be significantly reversed when using TNF-*α* synthesis inhibitors, suggesting that TNF-*α* is an important mediator of neuronal dysfunction and cognitive impairment triggered by chronic neuroinflammation.

In our study, patients were divided into 4 segments based on the serum concentration of defined parameters IL-6 and TNF-*α*. Based on the result output, the number of POCD was significantly different in these four segments. With the increase of the concentration of these two inflammatory factors, the frequency of POCD increased significantly. Analysis of Pearson correlation indicated the positive correlation of IL-6 concentration with POCD, i.e., *r* = 0.689 and *P* = 0.043. Likewise, plasma TNF-*α* concentration was also significantly correlated with POCD, i.e., *r* = 0.711 and *P* = 0.038. Both IL-6 and TNF-*α* play important roles in neurocognitive function, and their increased concentrations are predictive of decreased cognitive function; similarly, it is seen that the concentrations of both proinflammatory factors increase when POCD occurs. Concluding all, IL-6 and TNF-*α* concentrations were significantly correlated with the POCD values. The results of this trial further proved the validity of this theory.

Dexmedetomidine is the most discriminating and selective alpha-2 adrenergic receptor agonist. The most common uses of this receptor are sedation, narcotic analgesia, and anxiolysis. In this trial, the incidence of POCD was reduced from 21.31% to 9.2% both in the control and experimental group, respectively. The anti-inflammatory effect of dexmedetomidine has been found in recent years and may have a good protective effect on humans. There may be three ways for it to exert its anti-inflammatory effect [14,15]: (1) it activates the central a-Z receptor, inhibits the activity of sympathetic nerves, activates the anti-inflammatory pathway of cholinergic nerves, and reduces the level of proinflammatory factors. (2) It inhibits macrophages and reduces the secretion of tissue necrotizing factor *α*. (3) It reduces the concentration of IL-6 and TNF-*α* by gene regulation of kappa-B. This trial is concluded; dexmedetomidine reportedly reduced the increased concentration levels of IL-6 and TNF-*α* in the experimental group, which proved its anti-inflammatory effect. At the same time, dexmedetomidine has a protective effect on brain tissue. Some studies [16] have shown that dexmedetomidine can improve the oxygen metabolism in areas of cerebral hypoxia-reperfusion damage in rats and reduce the area of necrotic foci. A number of studies [17] at home and abroad showed that the postoperative MMSE score of the observational group is markedly lower than the dexmedetomidine intervention group, and the TNF-*α* and IL-6 levels and the incidence of postoperative POCD are markedly lower than those reported in the control group. The above results suggest that dexmedetomidine used for surgery in elderly patients can significantly improve patients' MMSE scores and minimize the incidence of early postsurgical cognitive dysfunction. The diagnosis of POCD still relies mainly on neuropsychological tests. The MMSE score is a simple, easy, and most influential screening tool for determining cognitive function. Therefore, in this study, the score was used, while the test was administered by the same specialized anesthesiologist at a fixed time, and the test details were explained to the patient before the test to minimize the possible influencing factors related to the test.

The incidence of postoperative POCD in the control group was 26.7% in this study, and the MMSE score increased and the incidence of POCD decreased after dexmedetomidine pretreatment, suggesting that dexmedetomidine pretreatment helps to prevent the occurrence of postoperative POCD in elderly patients with general anesthesia. The mechanism may be related to the ability of dexmedetomidine pretreatment to reduce the occurrence of inflammatory immunity and decrease the damage to the central nervous system of the organism.

## 5. Conclusion

1. Dexmedetomidine reduces the incidence of postoperative POCD in elderly patients.
2. Dexmedetomidine significantly reduces the increase in the postsurgical interleukin 6 and tissue necrotizing factor *α*.
3. The increase of interleukin 6 and tissue necrotizing factor *α* after surgery is significantly correlated with the increase of POCD.

## Figures and Tables

**Table 1:** Comparison of general data and intraoperative conditions of each indicator between two groups of patients (*χ*‾ ± *s*).

Groups	No. of cases	Age	Gender (M/F)	Weight (kg)	ASA grade (cases, II/III)	Education (years)	Operative time (min)	Bleeding volume (ml)	Sufentanil dosage (*μ*g)	Remifentanil dosage (mg)	Isoproterenol dosage (mg)
HC	87	71.4 ± 4.9	56/31	67 ± 8	71/16	10 ± 4	168 ± 53	406 ± 142	30.3 ± 3.8	2.38 ± 0.61	1485 ± 238
HS	87	70.6 ± 4.2	58/29	69 ± 8	76/11	11 ± 4	170 ± 48	428 ± 166	31.6 ± 4.2	2.51 ± 0.65	1533 ± 264

**Table 2:** TNF-*α* and IL-6 changes of serum concentrations of both groups (*n* = 30).

Indicators	Groups	Preoperative (T0)	Postoperative (T1h)
TNF-*α*（ng/L） HS	HC	46.20 ± 9.42	75.74 ± 10.39^*∗*^
	HS	45.28 ± 8.99^*∗*^	64.82 ± 9.71^*∗∗∗*^
IL-6（ng/L）	HC	51.02 ± 10.19	86.48 ± 13.51^*∗*^
	HS	49.44 ± 9.25^#^	69.04 ± 12.14^*∗∗∗*^

^*∗*^*P* < 0.05 indicates comparing postoperative with preoperative, ^*∗∗*^*P* < 0.05 indicates comparing both experimental and control group, and^#^ indicates *P* > 0.05 when comparing both experimental and control group.

**Table 3:** Comparing Mini-Mental State Examination (MMSE) scores and incidence of postoperative POCD between two groups of patients at different time points (scores, *χ*‾± *s*).

Groups	No. of cases	MMSE score		Incidence of POCD (cases (%))
		Preoperative （T10）	Postoperative T1（1d）	
HC	87	25.8 ± 0.8	25.6 ± 1.1^*∗*^	8(9.2)
HS	87	26.1 ± 0.7	22.2 ± 1.9^*∗∗∗*^	13 (21.3)^*∗*^
*P* values		0.86	0.04	0.038

^*∗*^*P* < 0.05 indicates comparing postoperative and preoperative and ^*∗∗*^*P* < 0.05 indicates comparing both experimental and control group.

**Table 4:** The cases of POCD in the data segment of the two proinflammatory factor quartiles.

Grade	No. of cases	IL-6 (ng/ml)	Incidence of POCD (cases (%))
Q1	22	57.96 (±10.06)	0 (0.00)
Q2	22	65.27 (±10.62)	1 (4.55)
Q3	22	70.34 (±11.82)	2 (9.09)
Q4	21	83.24 (±14.82)	5 (22.73)

**Table 5:** With the increase in the level of IL-6 concentration, the number of POCD increases significantly (*P* < 0.05).

Grade	No. of cases	TNF-*α* (ng/ml)	Incidence of POCD (cases (%))
Q1	22	55.28 (±11.27)	0 (0.00)
Q2	22	61.94 (±10.72)	1 (4.55)
Q3	22	66.18 (±11.71)	2 (9.09)
Q4	21	76.41 (±14.20)	5 (22.73)

## Data Availability

The data used to support the findings of this study are available from the corresponding author upon request.
